# Fully Convolutional Neural Network Deep Learning Model Fully in Patients with Type 2 Diabetes Complicated with Peripheral Neuropathy by High-Frequency Ultrasound Image

This article has been retracted.

**DOI:** 10.1155/2022/5466173

**Published:** 2022-03-24

**Authors:** Xiaoqiang Liu, Hongyan Zhou, Zhaoyun Wang, Xiaoli Liu, Xin Li, Chen Nie, Yang Li

**Affiliations:** ^1^Department of Ultrasound, The Second Hospital of Dalian Medical University, Dalian City, 116027 Liaoning Province, China; ^2^Department of Wound Repair, The Second Hospital of Dalian Medical University, Dalian City, 116027 Liaoning Province, China; ^3^Department of Respiratory, The Second Hospital of Dalian Medical University, Dalian City, 116027 Liaoning Province, China; ^4^Department of Radiology, The Second Hospital of Dalian Medical University, Dalian City, 116027 Liaoning Province, China; ^5^Department of Neurology, The Second Hospital of Dalian Medical University, Dalian City, 116027 Liaoning Province, China

## Abstract

This study was aimed at exploring the diagnostic value of high-frequency ultrasound imaging based on a fully convolutional neural network (FCN) for peripheral neuropathy in patients with type 2 diabetes (T2D). A total of 70 patients with T2D mellitus were selected and divided into a lesion group (*n* = 31) and a nonlesion group (*n* = 39) according to the type of peripheral neuropathy. In addition, 30 healthy people were used as controls. Hypervoxel-based and FCN-based high-frequency ultrasound images were used to examine the three groups of patients to evaluate their diagnostic performance and to compare the changes of peripheral nerves and ultrasound characteristics. The results showed that the Dice coefficient (92.7) and mean intersection over union (mIOU) (82.6) of the proposed algorithm after image segmentation were the largest, and the Hausdorff distance (7.6) and absolute volume difference (AVD) (8.9) were the smallest. The high-frequency ultrasound based on the segmentation algorithm showed higher diagnostic accuracy (94.0% vs. 86.0%), sensitivity (87.1% vs. 67.7%), specificity (97.1% vs. 94.2%), positive predictive value (93.1% vs. 86.7%), and negative predictive value (94.4% vs. 84.0%) (*P* < 0.05). There were significant differences in the detection values of the three major nerve segments of the upper limbs in the control group, the lesion group, and the nonlesion group (*P* < 0.05). Compared with the nonlesion group, the patients in the lesion group were more likely to have reduced nerve bundle echo, blurred reticular structure, thickened epineurium, and unclear borders of adjacent tissues (*P* < 0.05). In summary, the high-frequency ultrasound processed by the algorithm proposed in this study showed a high diagnostic value for peripheral neuropathy in T2D patients, and high-frequency ultrasound can be used to evaluate the morphological changes of peripheral nerves in T2D patients.

## 1. Introduction

Diabetes with peripheral neuropathy (PN) is one of the common chronic complications of diabetes [1]. The cause is that long-term high blood sugar causes continuous damage to peripheral nerves, which makes the peripheral nerves feel abnormal. Generally, it mainly damages the sense of temperature and pain, and the damage to the motor nerves is mild. Diabetes with PN, together with diabetic nephropathy and diabetic retinopathy, constitute the diabetic triad [2, 3]. The main clinical manifestations of the patient are the symmetry of the distal peripheral skin with coldness, tingling itching, and ant-walking sensation; sensory motivation disorders will also appear on the tip of the tongue; and the patient may also fall easily [4]. Type 2 diabetes (T2D) combined with PN (T2DPN) is generally seen in patients with a history of diabetes for more than 5 years, and patients with poor blood sugar control usually have PN [5–7]. The first clinical manifestation is abnormal sensation, which mainly manifests as numbness in the hands and feet, abnormal sensation, such as acupuncture-like sensation, ant-walking sensation, itching sensation, or hyperalgesia [8]. This numbness is generally symmetrical, starting from the distal end, and it is more common in the part of wearing socks or wearing gloves, so it is also called gloves or socks-like paresthesia in clinical practice [9]. In some patients, the muscles of both lower limbs are atrophy, especially the muscle atrophy between the tendons of the feet is more obvious [10].

For patients with T2D, early diagnosis and timely treatment are the basic measures to prevent diabetic neuropathy. At present, there are many ways to clinically check diabetic PN, such as nerve conduction velocity test and quantitative sensory test. However, these two tests all required specialist operations and are time-consuming, laborious, and costly, so it is limited in large-scale screening and routine examinations in diabetes clinics [11–13]. Clinical studies have shown that high-frequency ultrasound can clearly display the condition of peripheral nerves and accurately provide information on the course, distribution, echo, and anatomical relationship of surrounding tissues [14]. In recent years, high-frequency ultrasound has been widely used in the display of normal neural structures, the diagnosis of neuropathy, and the identification of tumors inside and outside the nerves [15, 16]. However, there are few studies on its diagnostic value in T2D mellitus with lower extremity peripheral neuropathy, and further research is needed.

The lesions in high-frequency ultrasound images need to be reviewed manually, which often leads to errors in diagnosis due to subjective awareness. Therefore, artificial intelligence segmentation algorithms are applied. The fully convolutional neural network deep learning model (FCNN-DL model) [17] was applied to systematically and standardized process the images or sounds by learning the internal laws and representation levels of sample data to improve the recognizability of imaging, aimed at improving the accuracy and clarity of the imaging results. In addition, the DCNN algorithm shows better application recognition performance in large-scale natural image datasets, realizing the structure of layer-by-layer hierarchical learning from the original pixels of the image [18].

Based on this, high-frequency ultrasound imaging technology based on the combination of FCN and supervoxel model would be used to diagnose patients with T2D complicated with peripheral neuropathy, and the diagnostic value of peripheral neuropathy before and after treatment was compared. It is aimed at improving the clinical application effect of ultrasound imaging in the diagnosis of peripheral neuropathy in diabetic patients and provide a reasonable reference for its diagnosis and treatment.

## 2. Data and Methods

### 2.1. Basic Data

Seventy patients with type 2 diabetes admitted to hospital from June 2019 to March 2020 were selected as the research subjects, including 36 males and 34 females. They were 36-79 years old, with an average age of 59.02 ± 1.24 years old. The course of the disease was 2-24 years, with an average of 13.4 ± 1.3 years, including 31 patients with the course of the disease shorter than 10 years (14 were males and 17 were females), 39 cases with the course of the disease longer than 10 years (18 were males and 21 were females). Patients were divided into a lesion group (*n* = 31) and a nonlesion group (*n* = 39) according to whether they had peripheral neuropathy or not. In addition, 30 healthy subjects during the same period were selected as the control group, including 14 males and 16 females. High-frequency ultrasound images based on supervoxel and FCN were used to examine the three groups of patients to evaluate their diagnostic performance and to compare and analyze the changes of peripheral nerves and ultrasound characteristics. The informed consent of all patients was obtained, and this study had been approved by the medical ethics committee of hospital.

Inclusion criteria are as follows: patients who met the diagnostic criteria with reference to the relevant diagnostic criteria of T2DPN in the diagnostic criteria of diabetes, patients who were confirmed with T2D through various biochemical tests, patients with complete clinical data, and patients whose family members know and sign the informed consent.

Exclusion criteria are as follows: patients with a history of relevant surgery; patients with other types of diabetes; patients with a history of malignancy; those with other serious diseases; those with immune system disorders; patients with allergies; those with poor adherence to the study; patients with a history of hypertension, coronary heart disease (CHD), and neuropathy; and patients with no positive signs on neurological examination.

### 2.2. Methods

#### 2.2.1. Construction of FCN

FCN implements pixel-level classification, which is mainly based on the traditional convolutional neural network model (CNN) with the following adjustments. Firstly, the convolutional layer was used to replace the fully connected layer in the traditional CNN model. This effectively relieved the display of the input image size by the fully connected layer and realized the simultaneous prediction of multiple pixels, which effectively reduced the computational complexity of the model. Secondly, the upsampling process had been added. This guaranteed the size of the output image. Thirdly, a cross-layer connection structure was used, which solved rough segmentation caused by deconvolution. The basic structure of the FCN model and the CNN model was shown in Figure 1.

In this study, an end-to-end CNN model fusion 3D supervoxel method was proposed for image segmentation. The basic structure of the model was shown in Figure 2.

The FCN model in this image was mainly composed of convolutional layer, BN layer, and ReLU. The pooling window size of the pooling layer was 3 × 3, the step size was set to 2, and the loss function used by the softmax layer as shown in the following equation:

(1) $$\begin{array}{c} \text{Loss}=-\overset{x}{\underset{i}{\sum }}\hat{u_{n}}\log f\left(z_{i}\right). \end{array}$$

In the above equation, $\hat{u}$ was the label value, and *f*(*z*_*i*_) referred to the probability that the sample belongs to different categories.

In this study, the SLIC supervoxel algorithm was adopted for image segmentation. It was assumed that the spatial position of a pixel in the five-dimensional space was (*a*_*i*_, *b*_*i*_, *c*_*i*_, *d*_*i*_, *e*_*i*_), and the position of the sample in the LAB color space was expressed as (*a*_*i*_, *b*_*i*_, *c*_*i*_); then, the position of the cluster center can be expressed as (*a*_*j*_, *b*_*j*_, *c*_*j*_, *d*_*j*_, *e*_*j*_).

At this time, the color distance from the *i*th pixel to the *j*th cluster center was expressed as below equation:

(2) $$\begin{array}{c} D_{abc}=\sqrt{{\left(a_{j}-a_{i}\right)}^{2}+{\left(b_{j}-b_{i}\right)}^{2}+{\left(c_{j}-c_{i}\right)}^{2}}. \end{array}$$

The spatial distance from the *i*th pixel to the *j*th cluster center was given as follows:

(3) $$\begin{array}{c} D_{de}=\sqrt{{\left(d_{j}-d_{i}\right)}^{2}+{\left(e_{j}-e_{i}\right)}^{2}}. \end{array}$$

The color distance and the space distance were normalized, and the calculation equation after processing was as follows:

(4) $$\begin{array}{c} D^{\sim }=\sqrt{{\left(\frac{D_{abc}}{Lc}\right)}^{2}+{\left(\frac{D_{de}}{Ls}\right)}^{2}}. \end{array}$$

In the above equation (4), *Lc* = *m* and $Ls=\sqrt{L/k}$.

#### 2.2.2. HFUS Examination

The subjects all were performed with HFUS examination based on FCNN-DL model. After 15 minutes in a quiet state, the color ultrasound diagnostic apparatus was applied for examination. The frequency of the probe was 8-10 MHz. The specific inspection method was as follows. The patient was assisted to choose the prone position with fully exposed legs. The examination was started from the thigh base downwards the ankle; the cross-section was scanned firstly, and then, the probe was rotated 90 degrees to scan the longitudinal section to show the main nerves of the lower limbs, including sciatic nerve, common peroneal nerve, tibial nerve, common peroneal nerve, and tibial nerve.

#### 2.2.3. Image Processing

The image data were normalized. The methods commonly used for data normalization processing included Min-Max and *Z*-score normalization. In this study, the Min-Max normalization method was used to normalize high-frequency ultrasound images. The calculation equation of this method was as follows:

(5) $$\begin{array}{c} x^{\sim }=\frac{\left(x-x_{\min}\right)}{\left(x_{\max}-x_{\min}\right)}. \end{array}$$

In the above equation, *x*^~^ was the normalized data, *x*_min_ was the minimum value in the pixel set, and *x*_max_ referred to the maximum value in the pixel set.

#### 2.2.4. Evaluation Indicators

In this study, the indicators Dice similarity, mean intersection over union (mIOU), Hausdorff distance, and absolute volume difference (AVD) were adopted to compare the effects of algorithms in processing image data. The calculation equations for different indicators were given as follows:

(6) $$\begin{array}{c} \text{Dice}=\frac{2\times \text{TP}}{\left(\text{TP}+\text{FN}\right)+\left(\text{TP}+\text{FP}\right)}. \end{array}$$

In the above equations, TP was true positive, FP referred to false positive, TN was true negative, and FN represented false negative.

(7) $$\begin{array}{c} \text{mIOU}=\frac{1}{n}\overset{n}{\underset{i=1}{\sum }}{\left(\frac{TP}{TP+FN+FP}\right)}_{i} \end{array}$$

In the above equation (7), IOU was within 0 ~ 1, and *n* was the number of classification.

(8) $$\begin{array}{c} \text{Hausdorff}=\max\left[\max_{a\in S}\min_{b\in GT}\left\|a-b\right\|,\max_{b\in G\text{T}}\min_{a\in S}\left\|a-b\right\|\right] \end{array}$$

Hausdorff distance was used to measure the maximum distance of the surface in space. The smaller the value, the better the segmentation effect.

(9) $$\begin{array}{c} \text{AVD}=\frac{\left|{\text{V}}_{\text{S}}-{\text{V}}_{\text{GT}}\right|}{{\text{V}}_{\text{GT}}}. \end{array}$$

In the above equation (9), *V*_*S*_ was the divided volume, and *V*_GT_ referred to the real volume.

### 2.3. Statistical Analysis

The collected data were sorted, summarized, and analyzed by SPSS 23.0. Measurement data were expressed as mean ± standard deviation ($\bar{x}\pm s$), single sample data was tested using the *t*-test; count data was tested by *x*^2^ and expressed in the form of number of cases (%). *P* < 0.05 indicated that the difference was statistically significant.

## 3. Results

### 3.1. Segmentation Algorithm Test Results

To verify the effectiveness of the proposed algorithm for high-frequency ultrasound image segmentation, it was compared with Snake [19], CNN [20], FCN8s [21], and SegNet [22] for segmentation of high-frequency images of patients with diabetes and peripheral neuropathy. The segmentation effect was shown in Figure 3. It can be observed that the Snake, CNN, and FCN8s algorithms only obtained the approximate outline of the lesion but failed to capture the detailed features of the lesion in place. SegNet and the algorithm proposed could better segment and process the boundary details of the lesion, but the algorithm proposed in showed a better processing effect on the details of tissue texture and boundary.

Then, the evaluation indicators Dice, miOU, Hausdorff, and AVD were adopted to quantitatively evaluate the segmentation effects of different algorithms, and the results were shown in Figure 4. It illustrated that the Dice and mIOU values after the Snake model divided the image were the smallest, while the Hausdorff and AVD values were the largest. On the contrary, the Dice and mIOU values of the proposed algorithm after image segmentation were the largest, while the Hausdorff and AVD values were the smallest.

### 3.2. Comparison of the Value of High-Frequency Ultrasound in Diagnosing Peripheral Neuropathy

100 samples were included for diagnostic value analysis. Among them, 69 patients had no peripheral nerve disease (30 healthy people, 39 patients with type 2 diabetes) and 31 patients with peripheral neuropathy (type 2 diabetes with peripheral neuropathy). The conventional high-frequency ultrasound and algorithm processing were adopted to compare the value of high-frequency ultrasound for disease diagnosis. Routine ultrasound diagnosed 21 true positive cases, 65 true negative cases, 4 false positive cases, and 10 false negative cases. Algorithm-based high-frequency ultrasound diagnosed 27 true positive cases, 67 true negative cases, 2 false positive cases, and 4 false negative cases. The diagnostic accuracy, sensitivity, specificity, positive predictive value, and negative predictive value of different methods were calculated, and the comparison of the diagnostic effects between the two groups of patients was shown in Figure 5. As it revealed, the value of algorithm-based high-frequency ultrasound diagnosis was significantly better than that of conventional ultrasound.

### 3.3. Comparison of Basic Patient Information

According to the diagnosis of high-frequency ultrasound and other data, among the 70 patients with type 2 diabetes, 31 had peripheral neuropathy, and 39 had no pathological changes. Therefore, the differences in the basic data of patients in the control group, the lesion group, and the nonlesion group were compared, and the results were shown in Table 1. There was no significant difference in the gender ratio and age of patients in three groups (*P* > 0.05). There was no significant difference in the course of disease data of patients between the lesion group and the lesion group (*P* > 0.05).

### 3.4. Distribution of Nerve Changes in Patients with Type 2 Diabetes and Peripheral Neuropathy

The nerve changes of patients with type 2 diabetes and peripheral neuropathy were compared. As given in Figure 6, the proportion of patients with thickening of the sciatic nerve was the largest (76%), followed by the thickening of the common peroneal nerve (21%), and the proportion of patients with the tibial nerve damage was the lowest (3%).

### 3.5. Comparison of Nerve Changes in each Group of Patients

The length (D1), width (D2), and cross-section area (CSA) of the cubital fossa (MN), the radial nerve running along the nerve groove (RN), and between the inner epicondyle and the olecranon (UN) of the patient were measured and calculated, and the results were given in Table 2. It can be observed that there were significant differences in MN-CSA, RN-D1, RN-CSA, UN-D1, and UN-CSA in the control group, the lesion group, and the nonlesion group, and the differences were statistically significant (*P* < 0.05).

### 3.6. Comparison of Ultrasound Features in Patients with Type 2 Diabetes

The changes in ultrasound characteristics of patients with type 2 diabetes were compared in the lesion and nonlesion groups, and the results were shown in Figure 7. Compared with patients with type 2 diabetes with no peripheral neuropathy, patients with type 2 diabetes with peripheral neuropathy were more likely to have reduced nerve bundle echo, blurred reticular structure, thickened epineurium, and unclear borders of adjacent tissues. And the difference was statistically significant (*P* < 0.05).

## 4. Discussion

The incidence of diabetic PN is increasing year by year, and it can be as high as 50% in western countries. Its pathogenesis is not yet fully understood, and it may be related to the metabolic disorders and abnormal microcirculation of the body and the body's own immune disorders [23–25]. Most of the disease has an insidious onset, and patients have no conscious symptoms at the beginning. When clinical symptoms appear, irreversible pathological changes have appeared in the peripheral nerves, which increases the risk and difficulty of clinical treatment and prognosis [26]. Therefore, early diagnosis and discovery of peripheral nerve damage are subjects of close clinical attention [27].

Although the current clinical examination methods are relatively reliable and objective examination methods, they have the disadvantages of being time-consuming, laborious, and high cost, so they cannot be used in large-scale screening and diabetic outpatient examinations [28]. An ultrasound can measure the cross-sectional area of each nerve, which can provide a morphological basis for the evaluation of the degree of PN in diabetic patients, and it can also provide information on changes in nerve stiffness. In this study, HFUS was used to examine the neurological conditions of T2DPN patients, and the FCNN-DL model was adopted to improve the pixel accuracy of ultrasound examination and better explore the diagnostic efficiency of the examination. The results of this study showed that the use of FCN fusion supervoxel model for the processing of high-frequency ultrasound images of patients had better segmentation effect than Snake, CNN, FCN8s, and SegNet models. Villa et al. [29] pointed out that the FCN-based method was superior to other algorithms in the segmentation effect of ultrasound images. Jiang et al. [30] also proposed that the FCN algorithm had a significant segmentation effect on CT images. Wang et al. [31] and See et al. [32] pointed out that the supervoxel segmentation effect had better advantages in their research. The above results suggest that the supervoxel and FCN algorithms have good application prospects in medical image segmentation, and give certain support to the results obtained in this work.

Subsequently, this study compared the difference in the diagnostic value of high-frequency ultrasound in patients with peripheral neuropathy before and after the algorithm processing. The results showed that compared with conventional ultrasound, after high-frequency ultrasound imaging processed by the algorithm proposed in this study was used for the diagnosis of peripheral neuropathy in patients, the accuracy (94.0%), sensitivity (87.1%), specificity (97.1%), positive predictive value (93.1%), and negative predictive value (94.4%) were significantly improved. It suggests that the ultrasound image processed by the algorithm can improve the diagnosis effect of the disease [33].

High-frequency ultrasound imaging technology can clearly and intuitively display the nerve distribution and morphology of peripheral neuropathy in patients with type 2 diabetes, which provides very valuable information for the clinical diagnosis and treatment of the disease [14]. This study subsequently compared the changes in neuromorphology in patients with type 2 diabetes and peripheral neuropathy. The results showed that the patient's elbow fossa's inner and upper cross-sectional area, the long diameter and cross-sectional area of the radial nerve along the nerve groove, and the long diameter and cross-sectional area between the inner epicondyle and the olecranon of the elbow were significantly different. The above indicators of diseased patients were significantly greater than those of nonsurgery patients and healthy people. Such results are consistent with the findings of Liu et al. [34]. In addition, it was found in this study that patients with type 2 diabetes and peripheral neuropathy had a significantly increased probability of reduced nerve bundle echo, blurred reticular structure, thickened epineurium, and unclear borders of adjacent tissues. This may be used because the blood sugar level in the body is too high, which makes the peripheral nerve carbohydrate components accumulate too much, the internal osmotic pressure of nerve cells increases, and the cells develop edema, which in turn increases the volume of nerve fiber bundles [35].

## 5. Summary

According to the above analysis, it was concluded that high-frequency ultrasound processed by the FCN fusion algorithm based on hypervoxel had a high diagnostic value for peripheral neuropathy in patients with T2D; and high-frequency ultrasound can be used to assess morphological changes in peripheral nerves in patients with T2D. However, due to the loss of reference image data in the research process, there were certain errors in the research results. Therefore, it was necessary to add image data to further complement the work. However, this work could reflect that the intelligent algorithm had good application prospects in clinical medical imaging assistance, showing higher clinical promotion value.

## Figures and Tables

**Figure 1:** The basic structure of CNN and FCN models. (a) The CNN model structure. (b) The FCN model structure. The red area referred to the segmentation boundary of neural tissue.

**Figure 2:** Flow for image segmentation algorithm.

**Figure 3:** The segmentation effect of high-frequency ultrasound images. The yellow area showed the segmentation boundary of the lesion part.

**Figure 4:** Comparison of quantitative indicators of image segmentation with different algorithm models. (a) The comparison of the Dice coefficient. (b) The comparison of the mIOU value. (c) The comparison of the Hausdorff value. (d) The comparison of the AVD value.

**Figure 5:** Comparison of the diagnostic value of peripheral neuropathy. Ac, Se, Sp, NPV, and PPV in the above figure referred to accuracy, sensitivity, specificity, negative predictive value, and positive predictive value, respectively.

**Figure 6:** Changes of peripheral nerve.

**Figure 7:** Comparison of ultrasound characteristics of patients with type 2 diabetes and peripheral neuropathy. ^∗^There was statistical significance compared with the lesion group (*P* < 0.05).

**Table 1:** Comparison of basic data of patients.

Item	Control group (*n* = 30)	Lesion group (*n* = 31)	Nonlesion group (*n* = 39)	*F* value	*P* value
Gender (cases (%))					
Males	14 (46.7)	16 (51.6)	20 (51.3)	0.949	0.261
Females	16 (53.3)	15 (48.4)	19 (48.7)		
Age (years old)	55.27 ± 2.8	57.62 ± 1.3	56.59 ± 1.4	1.337	0.148
Course of disease (years)	—	9.26 ± 1.3	9.58 ± 1.1	1.094	0.183

**Table 2:** Comparison of the measured values of the three major nerves of the upper limbs.

Parameter	Lesion group (*n* = 31)	Nonlesion group (*n* = 39)	Control group (*n* = 30)	*F* value	*P* value
MN					
D1	6.14 ± 0.32	5.63 ± 0.38	5.54 ± 0.45	2.096	0.094
D2	2.89 ± 0.31	2.57 ± 0.22	2.46 ± 0.25	2.105	0.098
CSA	13.89 ± 1.35	11.09 ± 1.21	10.76 ± 1.66	4.132	0.035^∗^
RN					
D1	5.64 ± 0.45	4.81 ± 0.33	4.67 ± 0.49	3.769	0.041^∗^
D2	2.76 ± 0.34	2.34 ± 0.25	2.29 ± 0.34	1.577	0.116
CSA	11.97 ± 1.75	9.07 ± 1.41	8.35 ± 1.55	5.549	0.009^∗^
UN					
D1	5.11 ± 0.45	4.46 ± 0.36	4.29 ± 0.49	3.988	0.032^∗^
D2	2.74 ± 0.46	2.72 ± 0.25	2.73 ± 0.49	0.512	0.356
CSA	10.98 ± 2.27	7.88 ± 1.09	7.75 ± 1.67	4.077	0.038^∗^

Note: ^∗^the comparison was statistically significant (*P* < 0.05).

## Data Availability

The data used to support the findings of this study are available from the corresponding author upon request.
